# A Novel Computational Tool for the Fractional-Order Special Functions Arising from Modeling Scientific Phenomena via Abu-Shady–Kaabar Fractional Derivative

**DOI:** 10.1155/2022/2138775

**Published:** 2022-07-22

**Authors:** M. Abu-Shady, Mohammed K. A. Kaabar

**Affiliations:** ^1^Department of Mathematics and Computer Science, Faculty of Science, Menoufia University, Egypt; ^2^Gofa Camp, Near Gofa Industrial College and German Adebabay, Nifas Silk-Lafto, 26649 Addis Ababa, Ethiopia; ^3^Institute of Mathematical Sciences, Faculty of Science, University of Malaya, Kuala Lumpur 50603, Malaysia

## Abstract

Recently, a generalized fractional derivative formulation, known as Abu-Shady–Kaabar fractional derivative, is studied in detail which produces satisfactory results that are consistent with conventional definitions of fractional derivative such as Caputo and Riemann-Liouville. To derive the fractional forms of special functions, the generalized fractional derivative is used. The findings demonstrate that the current findings are compatible with Caputo findings. In addition, the fractional solution to the Bessel equation is found. While modeling phenomena in engineering, physical, and health sciences, special functions can be encountered in most modeling scenarios related to electromagnetic waves, hydrodynamics, and other related models. Therefore, there is a need for a computational tool for computing special functions in the sense of fractional calculus. This tool provides a straightforward technique for some fractional-order special functions while modeling these scientific phenomena in science, medicine, and engineering.

## 1. Introduction

Fractional derivatives calculus is a significant theorem that is naturally extended from ordinary derivatives and has increased in popularity due to various applications. Several fractional-order models have appeared in various fields, such as physics [1–4] and engineering [5, 6]. Also, in [7, 8], 2D temporal–spatial fractional differential equations using extended fractional power series expansion is investigated, and the conformable-time-fractional Klein–Fock–Gordon equation is solved using the Kudryashov-expansion method to extract dual-wave solutions. In [9–11], the solutions of fractional gas dynamics equation, the nonisothermal flow of Williamson liquid over exponential surface, and the thermal radiative are considered by using a new fractional technique. Many studies use the time scales theory to deal with discrete formulations of fractional calculus [12–14]. There are several fractional derivative definitions in the literature, including Caputo (CP), Riemann-Liouville (RL), and Jumarie, although each has advantages and limitations. The most known one is the RL definition. For *m* − 1 ≤ *α* > *m*, the *α*-derivative of *g*(*s*) is expressed as

(1) $$\begin{array}{c} D^{RL}g\left(s\right)=\frac{1}{\Gamma \left(m-\alpha \right)}\frac{d^{m}}{dx^{m}}\int_{b}^{\infty }\frac{g\left(x\right)}{{\left(s-x\right)}^{\left(\alpha -m+1\right)}}dx, \end{array}$$

In the CP one, for *m* − 1 ≤ *α* > *m*, the *α*-derivative of *g*(*s*) is written as:

(2) $$\begin{array}{c} D^{CP}g\left(s\right)=\frac{1}{\Gamma \left(m-\alpha \right)}\int_{b}^{\infty }\frac{d^{m}g\left(x\right)/dx^{m}}{{\left(s-x\right)}^{\left(\alpha -m+1\right)}}dx. \end{array}$$

In [15], the conformable derivative (CD) is simply proposed by basically relying on the limit definition of the derivative.

(3) $$\begin{array}{c} D^{CD}g\left(s\right)=\underset{\delta ⟶0}{\lim}\frac{g\left(s+\delta s^{1-\alpha }\right)-g\left(s\right)}{\delta }. \end{array}$$

The CD has some advantages by satisfying some properties that are not verified in RL and CP definitions; however, in [16], the author proved that CD cannot have suitable results comparing with the good results using CP for some certain functions.

Recently, Abu-Shady and Kaabar introduced the generalized fractional derivative (GFD) that gives the compatible results with classical definitions such as RL and CP definitions. We give in the following section the basic definition including related theorems which are given in detail in [17]

(4) $$\begin{array}{c} D^{GFD}g\left(s\right)=\underset{\delta ⟶0}{\lim}\frac{g\left(s+\left(\Gamma \left(\gamma \right)/\Gamma \left(\gamma -\alpha +1\right)\right)\delta s^{1-\alpha }\right)-g\left(s\right)}{\delta };\gamma >-1,\gamma \in R^{+}. \end{array}$$

This work aims to apply the generalized fractional derivative for some special functions and gives the solution of Bessel equation in the fractional form which is essential in studying of physics science, engineering science, and health science. The motivation of the paper is given as a simple technique for the fractional special functions using GFD.

The work consists of four sections: Some fundamental definitions and theorems are introduced in Section 2. Some applications are presented for some special functions in Section 3. This work is concluded in Section 4.

## 2. Preliminaries

**Definition 1 .**

Given a function *g* : (0, ∞)⟶*R*, the GFD of order 0 < *α* ≤ 1 of *g*(*s*) at *s* > 0 is expressed as

(5) $$\begin{array}{c} D^{GFD}g\left(s\right)=\underset{\delta ⟶0}{\lim}\frac{g\left(s+\left(\Gamma \left(\gamma \right)/\Gamma \left(\gamma -\alpha +1\right)\right)\delta s^{1-\alpha }\right)-g\left(s\right)}{\delta };\gamma >-1,\gamma \in R^{+}, \end{array}$$

and the GFD at zero is *D*^*GFD*^*g*(0) = lim_*δ*⟶0_*D*^*GFD*^*g*(*s*).

**Theorem 1 .**

If *g*(*s*) is *α*−differentiable function(*Df*), then

(6) $$\begin{array}{c} D^{GFD}g\left(s\right)=\left(\Gamma \left(\gamma \right)/\Gamma \left(\gamma -\alpha +1\right)\right)s^{1-\alpha }\left(dg\left(s\right)/ds\right);\gamma >-1,\gamma \in R^{+}. \end{array}$$

**Theorem 2 .**

For a function derivative of *f*(*s*) = *s*^*l*^, *l*  ∈ *R*^+^, we obtain

(7) $$\begin{array}{c} D^{\alpha }D^{\gamma }s^{l}=D^{\alpha +\gamma }s^{l}. \end{array}$$

**Theorem 3 .**

For a Df: *f*(*s*) that expands about a point ∋*f*(*s*) = ∑_*k*=0_^∞^(*f*^*k*^(0)/*k*!)*s*^*k*^, the following is proven:

(8) $$\begin{array}{c} D^{\alpha }D^{\gamma }f\left(s\right)=D^{\alpha +\gamma }f\left(s\right). \end{array}$$

**Theorem 4 .**

Let *α*∈(0, 1], *H* and *W* are *α*-Dfs, then

(9) $$\begin{array}{c} \left(i\right)D^{GFD}\left(HW\right)=HD^{GFD}\left(W\right)+WD^{GFD}\left(H\right),\\ \left(ii\right)D^{GFD}\left(\frac{H}{W}\right)=\frac{WD^{GFD}\left(H\right)-HD^{GFD}\left(W\right)}{W^{2}}. \end{array}$$

## 3. Maclaurin's Series of Some Special Functions in the Fractional Forms

### 3.1. Natural Logarithm

(10) $$\begin{array}{c} 1-{\left(1-x\right)}^{n}=-\overset{\infty }{\underset{n=1}{\sum }}\frac{x^{n}}{n},\\ D^{GFD}{\left(1-x\right)}^{n}=-\overset{\infty }{\underset{n=1}{\sum }}\frac{1}{n}D^{GFD}x^{n}, \end{array}$$

from Ref. [17], we proved that

(11) $$\begin{array}{c} D^{GFD}x^{n}=\frac{\Gamma \left(n+1\right)}{\Gamma \left(n-\alpha +1\right)}x^{n-\alpha },\\ D^{GFD}x^{n}=D^{CP}x^{n}, \end{array}$$

therefore

(12) $$\begin{array}{c} D^{GFD}{\left(1-x\right)}^{n}=-\overset{\infty }{\underset{n=1}{\sum }}\frac{1}{n}D^{CP}x^{n},\\ D^{GFD}{\left(1-x\right)}^{n}=D^{CP}\left(-\overset{\infty }{\underset{n=1}{\sum }}\frac{1}{n}x^{n}\right),\\ D^{GFD}{\left(1-x\right)}^{n}=D^{CP}{\left(1-x\right)}^{n}. \end{array}$$

Similarly,

2 − (1 + *x*)^*n*^ = −∑_*n*=1_^∞^(−1)^*n*^(*x*^*n*^/*n*), then the fractional form:

(13) $$\begin{array}{c} D^{GFD}{\left(1+x\right)}^{n}=-\overset{\infty }{\underset{n=1}{\sum }}\frac{{\left(-1\right)}^{n}}{n}D^{GFD}x^{n},\\ D^{GFD}{\left(1+x\right)}^{n}=-\overset{\infty }{\underset{n=1}{\sum }}\frac{{\left(-1\right)}^{n}}{n}D^{CP}x^{n},\\ D^{GFD}{\left(1+x\right)}^{n}=D^{CP}\left(-\overset{\infty }{\underset{n=1}{\sum }}\frac{{\left(-1\right)}^{n}}{n}x^{n}\right),\\ D^{GFD}{\left(1+x\right)}^{n}=D^{CP}{\left(1+x\right)}^{n}. \end{array}$$

### 3.2. Geometric Series

The geometric series and its derivatives have Maclaurin's series as follows:

(14) $$\begin{array}{c} f\left(x\right)=\frac{1}{1-x}=\overset{\infty }{\underset{n=0}{\sum }}x^{n},\\ D^{GFD}f\left(x\right)=D^{GFD}\left(\frac{1}{1-x}\right)=\overset{\infty }{\underset{n=0}{\sum }}D^{GFD}x^{n},\\ D^{GFD}f\left(x\right)=D^{GFD}x^{0}+\overset{\infty }{\underset{n=1}{\sum }}\frac{\Gamma \left(n+1\right)}{\Gamma \left(n-\alpha +1\right)}x^{n-\alpha },\\ D^{GFD}f\left(x\right)=D^{CP}\overset{\infty }{\underset{n=0}{\sum }}x^{n},\\ D^{GFD}f\left(x\right)=D^{CP}f\left(x\right). \end{array}$$

Its derivative

(15) $$\begin{array}{c} \frac{df\left(x\right)}{dx}=\frac{1}{{\left(1-x\right)}^{2}}=\overset{\infty }{\underset{n=1}{\sum }}nx^{n-1},\\ D^{GFD}\frac{df\left(x\right)}{dx}=D^{GFD}\left(\frac{1}{{\left(1-x\right)}^{2}}\right)=\overset{\infty }{\underset{n=1}{\sum }}nD^{GFD}x^{n-1},\\ D^{GFD}\frac{df\left(x\right)}{dx}=D^{GFD}x^{0}+\overset{\infty }{\underset{n=2}{\sum }}\frac{\Gamma \left(n\right)}{\Gamma \left(n-\alpha \right)}x^{n-\alpha -1},\\ D^{GFD}\frac{df\left(x\right)}{dx}=D^{CP}\left(\overset{\infty }{\underset{n=1}{\sum }}nx^{n-1}\right),\\ D^{GFD}\frac{df\left(x\right)}{dx}=D^{CP}\frac{df\left(x\right)}{dx}. \end{array}$$

### 3.3. Binomial Series

The binomial series is the power series as

(16) $$\begin{array}{c} {\left(1+x\right)}^{k}=\overset{\infty }{\underset{n=0}{\sum }}\left(\begin{array}{c} k\\ n \end{array}\right)x^{n},\\ D^{GFD}{\left(1cx\right)}^{k}=\overset{\infty }{\underset{n=0}{\sum }}\left(\begin{array}{c} k\\ n \end{array}\right)D^{GFD}x^{n},\\ D^{GFD}{\left(1+x\right)}^{k}=\overset{\infty }{\underset{n=0}{\sum }}\left(\begin{array}{c} k\\ n \end{array}\right)D^{CP}x^{n},\\ D^{GFD}{\left(1+x\right)}^{k}=D^{CP}\left(\overset{\infty }{\underset{n=0}{\sum }}\left(\begin{array}{c} k\\ n \end{array}\right)x^{n}\right),\\ D^{GFD}{\left(1+x\right)}^{k}=D^{CP}{\left(1+x\right)}^{k}, \end{array}$$

where $\left(\begin{array}{c} k\\ n \end{array}\right)=\prod \lim_{i=1}^{n}\left(\left(k-i+1\right)/i\right)$

### 3.4. Trigonometric Functions

We take some trigonometric functions where their inverses have the following Maclaurin's series:

(17) $$\begin{array}{c} \tan x=\overset{\infty }{\underset{n=1}{\sum }}\frac{B_{2n}{\left(-4\right)}^{n}\left(1-4^{n}\right)}{\left(2n\right)!}x^{2n-1},\\ D^{GFD}\tan x=\overset{\infty }{\underset{n=1}{\sum }}\frac{B_{2n}{\left(-4\right)}^{n}\left(1-4^{n}\right)}{\left(2n\right)!}D^{GFD}x^{2n-1},\\ D^{GFD}\tan x=\overset{\infty }{\underset{n=1}{\sum }}\frac{B_{2n}{\left(-4\right)}^{n}\left(1-4^{n}\right)}{\left(2n\right)!}D^{CP}x^{2n-1},\\ D^{GFD}\tan x=D^{CP}\left(\overset{\infty }{\underset{n=1}{\sum }}\frac{B_{2n}{\left(-4\right)}^{n}\left(1-4^{n}\right)}{\left(2n\right)!}x^{2n-1}\right),\\ D^{GFD}\tan x=D^{CP}\tan x. \end{array}$$

Its inverse

(18) $$\begin{array}{c} \tan^{-1}x=\overset{\infty }{\underset{n=0}{\sum }}\frac{{\left(-1\right)}^{n}}{\left(2n+1\right)}x^{2n+1},\\ D^{GFD}\tan^{-1}x=\overset{\infty }{\underset{n=0}{\sum }}\frac{{\left(-1\right)}^{n}}{\left(2n+1\right)}D^{GFD}x^{2n+1},\\ D^{GFD}\tan^{-1}x=\overset{\infty }{\underset{n=0}{\sum }}\frac{{\left(-1\right)}^{n}}{\left(2n+1\right)}D^{CP}x^{2n+1},\\ D^{GFD}\tan^{-1}x=D^{CP}\left(\overset{\infty }{\underset{n=0}{\sum }}\frac{{\left(-1\right)}^{n}}{\left(2n+1\right)}x^{2n+1}\right),\\ D^{GFD}\tan^{-1}x=D^{CP}\tan^{-1}x. \end{array}$$

Also

(19) $$\begin{array}{c} \sin^{-1}x=\overset{\infty }{\underset{n=0}{\sum }}\frac{\left(2n\right)!}{4^{n}\left(n\right)!\left(2n+1\right)}x^{2n+1},\\ D^{GFD}\sin^{-1}x=\overset{\infty }{\underset{n=0}{\sum }}\frac{\left(2n\right)!}{4^{n}\left(n\right)!\left(2n+1\right)}D^{GFD}x^{2n+1},\\ D^{GFD}\sin^{-1}x=\overset{\infty }{\underset{n=0}{\sum }}\frac{\left(2n\right)!}{4^{n}\left(n\right)!\left(2n+1\right)}D^{CP}x^{2n+1},\\ D^{GFD}\sin^{-1}x=D^{CP}\left(\overset{\infty }{\underset{n=0}{\sum }}\frac{\left(2n\right)!}{4^{n}\left(n\right)!\left(2n+1\right)}x^{2n+1}\right),\\ D^{GFD}\sin^{-1}x=D^{CP}\sin^{-1}x. \end{array}$$

## 4. A Solution of Bessel Equation in the Fractional Form

Bessel equation [18] is given by:

(20) $$\begin{array}{c} x^{2}\frac{d^{2}y}{dx^{2}}+x\frac{dy}{dx}+\left(x^{2}-p^{2}\right)y=0, \end{array}$$

so, the fractional form of Bessel equation is written as in [19] as follows:

(21) $$\begin{array}{c} x^{2\alpha }D^{\alpha }D^{\alpha }y+\alpha_{1}D^{\alpha }y+{\left(\alpha_{1}\right)}^{2}\left(x^{2}-p^{2}\right)y=0, \end{array}$$

where *α*_1_ = (Γ(*γ*)/Γ(*γ* − *α* + 1))*α*, and

(22) $$\begin{array}{c} D^{\alpha }y\left(x\right)=\frac{\Gamma \left(\gamma \right)}{\Gamma \left(\gamma -\alpha +1\right)}x^{1-\alpha }\frac{dy}{dx}, \end{array}$$

(23) $$\begin{array}{c} D^{\alpha }D^{\alpha }y\left(x\right)={\left(\frac{\Gamma \left(\gamma \right)}{\Gamma \left(\gamma -\alpha +1\right)}\right)}^{2}\left[x^{2-2\alpha }\frac{d^{2}y}{dx^{2}}+\left(1-\alpha \right)x^{1-2\alpha }\frac{dy}{dx}\right]. \end{array}$$

At *α* = *γ* = 1, then Equation (21) is classical Bessel equation, and 0≺*α* ≤ 1 and 0≺*γ* ≤ 1. A fractional Frobenius series can be used to examine the following solution:

(24) $$\begin{array}{c} y=\overset{\infty }{\underset{n=0}{\sum }}c_{n}x^{\left(n+r\right)\alpha }, \end{array}$$

using the generalized fractional derivative from Equation (22)

(25) $$\begin{array}{c} D^{\alpha }y=\frac{\Gamma \left(\gamma \right)}{\Gamma \left(\gamma -\alpha +1\right)}\overset{\infty }{\underset{n=0}{\sum }}\left(n+r\right)\alpha c_{n}x^{\left(n+r-1\right)\alpha }, \end{array}$$

(26) $$\begin{array}{c} D^{\alpha }D^{\alpha }y={\left(\frac{\Gamma \left(\gamma \right)}{\Gamma \left(\gamma -\alpha +1\right)}\right)}^{2}\overset{\infty }{\underset{n=0}{\sum }}\left(n+r\right)\left(n+r-1\right)\alpha^{2}c_{n}x^{\left(n+r-2\right)\alpha }. \end{array}$$

substituting by Equations (24)–(26) into Equation (21)

(27) $$\begin{array}{c} \overset{\infty }{\underset{n=0}{\sum }}{\left(\alpha_{1}\right)}^{2}\left(n+r\right)\left(n+r-1\right)c_{n}x^{\left(n+r\right)\alpha }+\overset{\infty }{\underset{n=0}{\sum }}{\left(\alpha_{1}\right)}^{2}\left(n+r\right)c_{n}x^{\left(n+r\right)\alpha }+{\left(\alpha_{1}\right)}^{2}\left(x^{2}-p^{2}\right)\overset{\infty }{\underset{n=0}{\sum }}c_{n}x^{\left(n+r\right)\alpha }=0,\\ \left({\left(\alpha_{1}\right)}^{2}\left(r\right)\left(r-1\right)+{\left(\alpha_{1}\right)}^{2}r-{\left(\alpha_{1}\right)}^{2}p^{2}\right)c_{0}x^{r\alpha }+\left(\begin{array}{c} {\left(\alpha_{1}\right)}^{2}\left(r+1\right)\left(r\right)+{\left(\alpha_{1}\right)}^{2}\left(r+1\right)\\ -{\left(\alpha_{1}\right)}^{2}p^{2} \end{array}\right)c_{1}x^{\left(r+1\right)\alpha }+\overset{\infty }{\underset{n=2}{\sum }}\left[\left({\left(\alpha_{1}\right)}^{2}\left(n+r\right)\left(n+r-1\right)+{\left(\alpha_{1}\right)}^{2}\left(n+r\right)-{\left(\alpha_{1}\right)}^{2}p^{2}\right)c_{n}+{\left(\alpha_{1}\right)}^{2}c_{n-2}\right]x^{\left(n+r\right)\alpha }=0. \end{array}$$

If we define

(28) $$\begin{array}{c} L\left(r\right)={\left(\alpha_{1}\right)}^{2}\left(r\right)\left(r-1\right)+{\left(\alpha_{1}\right)}^{2}r-{\left(\alpha_{1}\right)}^{2}p^{2}, \end{array}$$

then we can Equation (21) as

(29) $$\begin{array}{c} L\left(r\right)c_{0}x^{r\alpha }+L\left(r+1\right)c_{1}x^{\left(r+1\right)\alpha }+\overset{\infty }{\underset{n=2}{\sum }}\left[L\left(r+n\right)c_{n}+{\left(\alpha_{1}\right)}^{2}c_{n-2}\right]x^{\left(n+r\right)\alpha }=0. \end{array}$$

If *c*_0_ ≠ 0, then

(30) $$\begin{array}{c} L\left(r\right)=0 \end{array}$$

and *α*_1_ ≠ 0, then

(31) $$\begin{array}{c} {\left(\alpha_{1}\right)}^{2}\left(r\right)\left(r-1\right)+{\left(\alpha_{1}\right)}^{2}r-{\left(\alpha_{1}\right)}^{2}p^{2}=0\Rightarrow r_{1}=p\text{or}r_{2}=-p \end{array}$$

Let us start with *p*0 case and obtain fractional Bessel equation solutions as follows:

For *r*_1_ = *p*, we get

(32) $$\begin{array}{c} L\left(p+1\right)c_{1}=0\Rightarrow \left(\left(2p+1\right)\right)c_{1}=0\Rightarrow c_{1}=0. \end{array}$$

In addition, the stated recurrence relation here is also accurate.

(33) $$\begin{array}{c} c_{2n}=-\frac{{\left(\alpha_{1}\right)}^{2}}{L\left(P+n\right)}c_{n-2}=-\frac{1}{n\left(P+n\right)}c_{n-2}\text{for }n\geq 2. \end{array}$$

Because *c*_1_ = 0 is an arbitrary constant, we can use the recurrence relation to find

(34) $$\begin{array}{c} c_{3}=c_{5}=\cdots =0. \end{array}$$

By using the recurrence relation, we have

(35) $$\begin{array}{c} c_{2n}=\frac{{\left(-1\right)}^{n}}{2^{n}n!\left(P+1\right)\left(P+2\right)\cdots \left(P+n\right)}c_{0}. \end{array}$$

As a result, the first solution of fractional Bessel Equation of order *p* is

(36) $$\begin{array}{c} y=\overset{\infty }{\underset{n=0}{\sum }}\frac{{\left(-1\right)}^{n}}{2^{n}n!\left(P+1\right)\left(P+2\right)\cdots \left(P+n\right)}c_{0}x^{\left(n\right)\alpha }, \end{array}$$

if taking *c*_0_ = *c*/Γ(*P* + 1) and the first solution of generalized fractional the Bessel equation of order *p*

(37) $$\begin{array}{c} y_{1}\left(x\right)=c\overset{\infty }{\underset{n=0}{\sum }}\frac{{\left(-1\right)}^{n}}{n!\Gamma \left(P+1\right)}{\left(\frac{x^{\alpha }}{2}\right)}^{2n+p} \end{array}$$

Besides, the Bessel function of order *p* is valid.

(38) $$\begin{array}{c} {\left(J_{\alpha }\right)}_{p}\left(x\right)=c\overset{\infty }{\underset{n=0}{\sum }}\frac{{\left(-1\right)}^{n}}{n!\Gamma \left(P+1\right)}{\left(\frac{x^{\alpha }}{2}\right)}^{2n+p}, \end{array}$$

for *r*_2_ = −*p*, the Bessel function of order *p*

(39) $$\begin{array}{c} {\left(J_{\alpha }\right)}_{p}\left(x\right)=c\overset{\infty }{\underset{n=0}{\sum }}\frac{{\left(-1\right)}^{n}}{n!\Gamma \left(P+1\right)}{\left(\frac{x^{\alpha }}{2}\right)}^{2n-p}. \end{array}$$

Equations (38) and (39) are compatible with results of [19].

## 5. Conclusion

The GFD formulation, known as Abu-Shady–Kaabar fractional derivative, is applied on the some special functions due to their importance while modeling systems in ocean engineering and science. We have proved that it is compatible with CP findings. Furthermore, the GFD provides the solution to the fractional Bessel equation. Thus, the GFD is simple and valid fractional definition which deals with some special functions that plays an essential role in physics, health sciences, and engineering fields.

## Data Availability

No data were used to support this study.
